RETRACTED

# MicroRNA-202 inhibits cell migration and invasion through targeting FGF2 and inactivating Wnt/β-catenin signaling in endometrial carcinoma

**DOI:** 10.1042/BSR20190680

**Published:** 2019-10-11

**Authors:** Ping Chen, Tianrong Xing, Qingdong Wang, Ai Liu, Haiping Liu, Yuhong Hu, Yanjia Ji, Ying Song, Dongwei Wang

**Affiliations:** 1 Department of Obstetrics and Gynecology, The First Affiliated Hospital of Jiamusi University, Heilongjiang Province 154002, P.R. China; 2 Department of Anesthesiology, The First Affiliated Hospital of Jiamusi University, Heilongjiang Province 154002, P.R. China; 3 Department of Gynaecology and Obstetrics, People’s Hospital of Zoucheng, Jining 273500, Shandong Province, P.R. China

**Keywords:** cell invasion, cell migration, endometrial carcinoma, FGF2, miR-202

## Abstract

Recently, many mircroRNAs (miRNAs) involved in the development and progression of cancer have been reported to regulate cell growth and metastasis, including microRNA-202 (miR-202). The purpose of the present study was to elucidate the effect of miR-202 on endometrial carcinoma (EC) cell migration and invasion. First, qRT-PCR showed that miR-202 was down-regulated in EC tissues, which was associated with poor prognosis in EC patients. Functionally, transwell assay indicated that miR-202 inhibited cell migration and invasion in EC cells. In addition, miR-202 also blocked epithelial–mesenchymal transition (EMT) through suppressing N-cadherin and Vimentin expressions and promoting E-cadherin expression. Moreover, the dual-luciferase reporter assay showed that fibroblast growth factor 2 (FGF2) is a direct target gene for miR-202 in EC cells. Furthermore, up-regulation of FGF2 attenuated the inhibitory effect of miR-202 on cell migration and invasion in EC. Besides that, miR-202 inactivated the Wnt/β-catenin signaling by suppressing β-catenin expression in EC. In conclusion, miR-202 inhibited cell migration and invasion by targeting FGF2 and inactivating the Wnt/β-catenin signaling in EC.

## Introduction

Endometrial cancer (EC) has become a major threat to women’s health and its incidence is increasing [1]. Fortunately, EC patients can get a good prognosis through surgery [2]. Although more than 70% of EC patients can be diagnosed early, up to 28% of EC patients will suffer local or distant metastases [3]. In addition, some EC patients have a risk of cancer recurrence and death, and those patients that relapse have a poor prognosis [4]. Effective treatments are still rare for advanced and relapsed EC patients, therefore, it is important to develop new EC treatment strategies.

Cell metastasis is important to the development of malignant tumors. Epithelial-mesenchymal transition (EMT) is an important regulatory mechanism driving cancer metastasis, including metastasis in EC [5]. Recently, there has been extensive investigation into the roles of mircroRNAs (miRNAs) in EMT and cell metastasis. For example, one study found that miR-101-3p attenuated the metastasis of glioblastoma cells by inhibiting EMT [6]. In contrast, miR-103 was found to promote metastasis and EMT by directly inhibiting the expression of LATS2 in hepatocellular carcinoma [7]. Similarly, specific functions of miRNAs have also been found in EC. MiR-23a was shown to inhibit EMT in EC via targeting SMAD3 [8], while miR-652 was reported to promote proliferation and metastasis of EC cells by regulating RORA expression [9]. MiR-202 may also play an important role in different cancers. For example, miR-202 suppressed cell proliferation in EC by targeting FOXR2 [10], and low miR-202 expression was shown to contribute to migration and invasion of esophageal squamous cell carcinoma cells [11]. However, whether miR-202 regulates EMT and cell migration and invasion in EC remains unknown.

RETRACTED

Fibroblast growth factor 2 (FGF2) is a member of the FGF family (which has 18 members: FGF1–FGF10 and FGF16–FGF23) [12] and is a potential miRNA target gene. It has been reported that FGF2 is involved in the regulation of cell metastasis and tumor formation [13]. Furthermore, up-regulation of FGF2 was identified in several human cancers, including glioblastoma, breast cancer and non-small-cell lung cancer (NSCLC) [14–16]. Previous studies also showed that FGF2 exerted its effect in cancers by interacting with some miRNAs. For example, miR-203 inhibited renal cancer cell migration, invasion and proliferation via FGF2 targeting [17]. Additionally, miR-195 suppressed the proliferation of colorectal cancer cells by targeting FGF2 and mediating Wnt/β-catenin signaling [18]. The Wnt/β-catenin pathway has been reported to be involved in the development of EC and is also regulated by miRNAs [19]. For instance, miR-373 promoted the development of EC by stimulating the Wnt/β-catenin pathway [20]. However, the role of FGF2 and its relationship with miR-202 is still unclear in EC.

Here, we investigated the function of miR-202 in EC, particularly whether miR-202 miR-202 regulates migration and invasion of EC cells. To further elucidate the regulatory mechanism of miR-202, the interaction between miR-202 and FGF2 was explored in EC cells. Additionally, we investigated the effect of miR-202 on β-catenin expression in EC. Understanding the function of miR-202 in EC may lead to new treatment strategies for EC.

## Materials and methods

### Clinical samples

Experimental EC tissues and normal specimens were obtained from 76 female EC patients in the first affiliated hospital of Jiamusi University and Zoucheng People’s Hospital. Based on the clinical pathological stage of EC, patients were classified as follows: 34 were stage I; 20 were stage II; 16 were stage III; and 6 were stage IV. All EC patients did not receive any treatment prior to surgery. All participants provided written informed consent before the study, and the Human Ethics Committee of the above three hospitals approved the present study.

RETRACTED

### Cell culture

Immortalized endometrial fibroblast cell T-HESCs (ATCC® CRL-4003™) and human EC cell lines HEC-1-B (ATCC® HTB-113™) and HEC-1-A (ATCC® HTB-112™) were purchased from ATCC (Manassas, VA, U.S.A.). These cells were cultured in DMEM medium (Invitrogen; Waltham, MA, U.S.A.) containing 10% fetal bovine serum (FBS), and incubated at 37°C in an atmosphere with 5% CO_2_.

### Cell transfection

MiR-202 mimics (sense: 5′-AGA GGU AUA GGG CAU GGG AA-3′, antisense: 5′-CCC AUG CCC UAU ACC UCU UU-3′), negative control (NC, sense: 5′-UUC UCC GAA CGU GUC ACG UTT-3′, antisense: 5′-ACG UGA CAC GUU CGG AGA ATT-3′) and miR-202 inhibitor (5′-UUC CCA UGC CCU AUA CCU CU-3′) or FGF2 plasmid (RiboBio Inc, GuangZhou, China) was severally transferred into HEC-1-B cells using Lipofectamine 2000 (Invitrogen, CA, U.S.A.). A sequence having no homology to humans was set as a NC.

### Quantitative RT-PCR

The extraction of total RNA was performed in EC tissues and cells using TRIzol reagent (Invitrogen, MA, U.S.A.). First-Strand cDNA Synthesis kits (Invitrogen) was used to obtain cDNA solution. Next, qRT-PCR assay was performed on Applied Biosystems 7500 detection system (Applied Bio-systems) using SYBR Prime Script RT-PCR kit (TaKaRa, Dalian, China). The expressions of miR-202 and FGF2 were evaluated by the 2^−ΔΔCq^ method using U6 and GAPDH as controls. The following primers were used: miR-202, forward 5′-CCT CCC AGG CTC ACG AGG CT-3′ and reverse 5′-GGT GCA GGT GCA CTG GTG CA-3′; U6, forward 5′-CAA AGT CAG TGC AGG TAG GCT TA-3′ and reverse 5′-AAC GCT TCA CGA ATT TGC GT-3′; FGF2, forward 5′-CCG TTA CCT GGC TAT GAA GG-3′ and reverse 5′-ACT GCC CAG TTC GTT TCA GT-3′; GAPDH, forward 5′-TTG ATG GCA ACA ATC TCC AC-3′ and reverse 5′-CGT CCC GTA GAC AAA ATG GT-3′.

### Western blot analysis

Protein samples were lysed using RIPA buffer (Beyotime, Shanghai, China). Protein concentration was measured using a BCA kit (Beyotime). The protein was then separated by 10% SDS/PAGE protein loading buffer. Next, the protein was transferred to PVDF membranes and incubated with primary antibodies (E-cadherin, N-cadherin, Vimentin, FGF2, β-catenin and GAPDH) overnight at 4°C. After washing, the protein was incubated with the corresponding secondary antibody for 1 h. Protein was detected using an Enhanced chemiluminescence solution (Pierce; Thermo Fisher Scientifc, Inc.) and protein images were obtained by FluorChem imaging system (Alpha Innotech, CA, U.S.A.).

RETRACTED

### Immunohistochemistry

The sections of paracancerous tissues were dewaxed, hydrated and washed twice with PBS for 5 min. After blocking with 5% goat serum (diluted in PBS), we incubated the cells with anti-FGF2 antibody at 37°C for 1–2 h. Then, the section was washed for three times with PBS for 5 min. Next, the section was incubated with the secondary antibody at 37°C for 1 h. After washing three times with PBS, DAB mixture was used for color development of this section. The section was washed, counterstained, dehydrated, transparentized and mounted. Images were captured using microscope.

### Transwell assay

Transwell assays were performed using 8-μm Transwell chambers (Corning Incorporated, NY, U.S.A.). Transwell chambers coated with Matrigel (BD Biosciences, NJ, U.S.A.) were used for cell invasion. However, cell migration was detected using Transwell chambers without BD. An upper chamber with HEC-1-B cells (5×10^4^/well) and a lower chamber containing a medium with 20% FBS were prepared. After 24 h, the cells were fixed and stained. Finally, migrated and invading cells were measured using an inverted microscope (Olympus Corporation, Tokyo, Japan).

### *In vitro* scratch assay

Each well of a 24-well plate was seeded with 800 μl HEC-1-B cell suspension (2×10^3^ cells/well) and incubated for 24 h at 37°C in an atmosphere containing 5% CO_2_. Once a confluent monolayer was formed, cells were serum-starved for 24 h and the cell monolayers were subsequently scratched using a 1000-μl pipette tip. Scratched cells were cultured in DMEM medium supplemented with 10% FBS for 24 h and observed under an inverted microscope (Olympus BX50; Tokyo, Japan; magnification, ×10). The migratory ability of the cells was assessed by comparing the respective repair distances.

### Dual-luciferase reporter gene assay

First, the 3′-UTR of wild or mutant type FGF2 was inserted into the pmirGLO luciferase reporter vector (Promega, U.S.A.). Next, HEC-1-B cells were transfected with the above luciferase vector and miR-202 mimics. After incubation of 48 h, luciferase activity was detected by a dual-luciferase reporter assay system (Promega, U.S.A.).

### Statistical analysis

All experiments were repeated three times independently. Data are shown as mean ± SD, which were analyzed using SPSS 19.0 and Graphpad Prism 6. Differences between groups were tested using χ^2^ test or ANOVA with Tukey’s post hoc test. Kaplan–Meier analysis with log-rank test was used to calculate survival differences. *P*<0.05 was considered to be significantly different.

RETRACTED

## Results

### Down-regulation of miR-202 was observed in EC

First, the mRNA expression of miR-202 was assessed in EC tissues by qRT-PCR. The results showed that the expression of miR-202 in EC tissues was lower than in normal tissues (Figure 1A). Next, the association between miR-202 expression and clinical features in EC patients was analyzed. We found that abnormal expression of miR-202 was closely related to FIGO stage or lymph node metastasis (Table 1). Furthermore, low miR-202 expression was associated with shorter overall survival in EC patients, suggesting that low miR-202 expression predicts poor prognosis in EC patients (Figure 1B). These results suggest that miR-202 may regulate the progression and prognosis of EC.

**Figure 1:** MiR-202 was down-regulated in EC tissues (**A**) The alternation of miR-202 expression in EC tissues. (**B**) Difference of overall survival between EC patients with high or low miR-202 expression. *P<0.05, **P<0.01.

**Table 1:** Relationship between miR-202 expression and their clinic-pathological characteristics of endometrial cancer patients

Characteristics	Cases	miR-202		*P*-value
		High	Low	
**Age (years)**				0.562
≥50	44	18	26	
<50	32	10	22	
**Pathology classification**				0.063
Well + Mod	50	15	35	
Poor	26	13	13	
**FIGO stages**				0.021*
I + II	54	20	34	
III + IV	22	8	14	
**Grade**				0.651
G1	30	5	25	
G2/3	46	23	23	
**Lymph node metastasis**				0.031*
Negative	42	6	36	
Positive	34	22	12	

Statistical analyses were performed by the χ2 test.

* *P*<0.05 was considered significant.

### MiR-202 inhibited cell migration and invasion in EC

Next, the expression level of miR-202 was measured in EC cell lines (HEC-1-B, HEC-1-A) and T-HESCs cells. Consistent with the above results, down-regulation of miR-202 was detected in HEC-1-B and HEC-1-A cells compared to T-HESCs cells (Figure 2A). HEC-1-B cells were selected for the further experiment. When the cell density reaches 70%, miR-202 mimics or inhibitor was transfected into HEC-1-B cells. The transfection efficiency was assessed using qRT-PCR. We found that miR-202 mimics enhanced the expression level of miR-202, while miR-202 inhibitor reduced its expression (Figure 2B). Functionally, overexpression of miR-202 was found to inhibit cell migration in HEC-1-B cells. In contrast, knockdown of miR-202 promoted HEC-1-B cell migration (Figure 2C). The scratch assay also showed that cell migration was inhibited by overexpression of miR-202 and promoted by down-regulation of miR-202 in HEC-1-B cells (Figure 2D). Similarly, miR-202 mimics inhibited HEC-1-B cell invasion, while miR-202 inhibitor promoted HEC-1-B cell invasion (Figure 2E). Briefly, miR-202 exerted an inhibitory effect on EC cell metastasis by inhibiting cell migration and invasion.

RETRACTED

**Figure 2:** MiR-202 suppressed cell metastasis in EC (**A**) MiR-202 expression in HEC-1-B, HEC-1-A and T-HESCs cell lines. (**B**) MiR-202 expression regulated by its mimics or inhibitor in HEC-1-B cells. (**C,D**) Cell migration regulated by miR-202 mimics or inhibitor was detected by Wound and Transwell assay. (**E**) Cell invasion regulated by miR-202 mimics or inhibitor in HEC-1-B cells. **P<0.01.

### MiR-202 inhibited EMT and inactivated Wnt/β-catenin signaling in EC

Furthermore, whether miR-202 regulates EMT and Wnt/β-catenin signaling was investigated in HEC-1-B cells. Overexpression of miR-202 was found to reduce expressions of N-cadherin and Vimentin and promote expression of E-cadherin in HEC-1-B cells. However, knockdown of miR-202 showed an opposite effect on their expressions (Figure 3). Besides that, the Wnt/β-catenin pathway is known to be involved in cell metastasis. Therefore, we detected the expression of β-catenin in HEC-1-B cells with miR-202 mimics or inhibitor. We found that the protein level of β-catenin was inhibited by miR-202 mimic and promoted by knockdown of miR-202 (Figure 3). Based on these results, we consider that miR-202 may be involved in EC cell metastasis by blocking EMT and suppressing β-catenin expression.

**Figure 3:** MiR-202 inhibited EMT and blocked Wnt/β-catenin pathway in EC The protein expressions of E-cadherin, N-cadherin, Vimentin and β-catenin regulated by miR-202 mimics or inhibitor in HEC-1-B cells

### FGF2 was a direct target of miR-202

Further, TargetScan (http://www.targetscan.org/) database was used to determine the target of miR-202 to explain its regulatory mechanism in EC. FGF2 was found to have a binding site with miR-202 (Figure 4A). Thus, we designed luciferase reporter assay to validate the above prediction. The results showed that miR-202 mimics reduced the luciferase activity of Wt-FGF2, but had no effect on Mut-FGF2 luciferase activity (Figure 4B). Furthermore, miR-202 was negatively correlated with FGF2 expression in EC tissues (R^2^ = 0.6597; Figure 4C). In addition, the alternation of FGF2 expression induced by miR-202 mimics or inhibitor was assessed in HEC-1-B cells. Consistently, overexpression of miR-202 decreased the mRNA and protein expression of FGF2, while miR-202 inhibitor promoted FGF2 expression in HEC-1-B cells (Figure 4D,E). Therefore, miR-202 was confirmed to directly target FGF2 and inhibit the expression of FGF2 in EC.

RETRACTED

**Figure 4:** FGF2 was a direct target of miR-202 (**A**) The binding sites between FGF2 with miR-202. (**B**) Luciferase reporter assay. (**C**) A negative correlation between miR-200 with FGF2 in EC tissues (**D,E**) MiR-202-mediated FGF2 expression in HEC-1-B cells. **P<0.01.

### Up-regulation of FGF2 impaired the suppressive effect of miR-202 in EC

Finally, mRNA expression of FGF2 was measured in EC tissues and cell lines. The results showed that FGF2 was up-regulated in EC tissues compared with normal tissues (Figure 5A,B). Similarly, up-regulation of FGF2 was also detected in HEC-1-B and HEC-1-A cells compared with T-HESCs cells (Figure 5C). To investigate the regulatory mechanism of miR-202 in EC, we transfected miR-202 mimics and FGF2 vector into HEC-1-B cells. Up-regulation of FGF2 was found to restore the decreased expression of FGF2 induced by miR-202 mimics (Figure 5D,E). Furthermore, overexpression of FGF2 also abolished the decreased expressions of N-cadherin, Vimentin and β-catenin and increased expression of E-cadherin caused by miR-202 mimics (Figure 5F). Functionally, transfection of FGF2 vector impaired miR-202-mediated inhibition of cell migration and invasion in EC cells (Figure 5G–J). These findings revealed that miR-202 inhibited cell migration and invasion by targeting FGF2 in EC.

**Figure 5:** Up-regulation of FGF2 impaired the inhibitory effect of miR-202 in EC (**A**) FGF2 mRNA expressions in EC tissues. (**B**) Expression of FGF2 in paracancerous tissues detected by immunohistochemistry and Western blot assay. (**C**) FGF2 expression in HEC-1-B, HEC-1-A and T-HESCs. (**D,E**) FGF2 expression in HEC-1-B cells with FGF2 vector and miR-202. (**F**) E-cadherin, N-cadherin, Vimentin and β-catenin expression in HEC-1-B cells with FGF2 vector and miR-202. (**G,I**) The detection of cell migration and invasion in HEC-1-B cells with FGF2 vector and miR-202 was assessed by Transwell assay. (**H,J**) Cell migration in HEC-1-B cells with FGF2 vector and miR-202 was detected by Wound assay. **P<0.01.

## Discussion

In recent years, miRNA has become a key player in the development of malignant tumors. Among them, many miRNAs have been found to be abnormally expressed in EC tissues, and such abnormal expression often leads to tumorigenesis. In those differentially expressed miRNAs, abnormal expression of miR-202 was found to be associated with the development of EC. In the present study, down-regulation of miR-202 was detected in EC tissues, which was associated with aggressive behaviors in EC patients. Functionally, miR-202 inhibited cell migration, invasion and EMT in EC. Furthermore, miR-202 inactivated the Wnt/β-catenin pathway by suppressing β-catenin expression in EC.

RETRACTED

Previous studies had reported that miR-202 was down-regulated in several cancers, including esophageal squamous cell carcinoma and pancreatic cancer [21,22], which was similar to our results. In addition, the inhibitory role of miR-202 was observed in breast cancer, gastric cancer and cervical cancer [23–25]. In particular, miR-202 was found to inhibit cell proliferation via inhibiting the expression of ARL5A in human colorectal carcinoma [26]. Similarly, miR-202 suppressed cell growth and metastasis in prostate cancer [27]. In the present study, the same inhibitory effect of miR-202 on cell migration and invasion was also identified in EC. Besides that, the Wnt/β-catenin pathway is involved in cell metastasis [28]. Moreover, it was found that the dysregulation of the Wnt/β-catenin pathway plays an important role in the development and progression of EC [29]. Here, the expression of β-catenin, as an important regulator of the Wnt/β-catenin pathway, was suppressed by overexpression of miR-202. It indicated that miR-202 inactivated the Wnt/β-catenin pathway in EC.

In present study, miR-202 was found to directly target FGF2 as well. And up-regulation of FGF2 attenuated the inhibitory effect of miR-202 in EC. It had been reported that FGF-2 could regulate cell proliferation and migration in human cancer [30]. Up-regulation of FGF2 and its carcinogenesis had been identified in esophageal cancer and osteosarcoma [31,32]. Furthermore, FGF2 was found to down-regulate the expression of E-cadherin in ovarian cancer [33]. In addition, the interaction between miRNAs and FGF2 was also investigated in other cancers. For instance, miR-646 suppressed osteosarcoma cell metastasis by inhibiting FGF2 expression [34]. MiR-195 inhibited EMT through suppressing FGF2 expression in prostate cancer [35]. In the current study, the relationship between miR-202 and FGF2 was also investigated in EC. Consistent with the above results, miR-202 also inhibited cell migration and invasion through targeting FGF2 in EC.

In conclusion, the expression of miR-202 was reduced in EC. Furthermore, miR-202 inhibited EC cell migration and invasion as well as EMT through targeting FGF2. Since miR-202 is able to inhibit EC cell metastasis, the alternation of miR-202 expression can be used as a diagnostic indicator for EC. Nevertheless, a more detailed study about the regulatory mechanism of miR-202 in EC pathogenesis still requires further clarification.

## Abbreviations

EC: endometrial carcinoma
EMT: epithelial–mesenchymal transition
FBS: fetal bovine serum
FGF2: fibroblast growth factor 2
miRNA: miRNA
NC: negative control
